RETRACTED

# Clinical Characteristics and Gene Mutation Analysis of Poststroke Epilepsy

**DOI:** 10.1155/2022/4801037

**Published:** 2022-08-29

**Authors:** Deju Shen, Yuqin Deng, Chunyan Lin, Jianshu Li, Xuehua Lin, Chaoning Zou

**Affiliations:** Department of Neurology, Longyan People Hospital, Longyan 364000, Fujian, China

## Abstract

Epilepsy is one of the most common brain disorders worldwide. Poststroke epilepsy (PSE) affects functional retrieval after stroke and brings considerable social values. A stroke occurs when the blood circulation to the brain fails, causing speech difficulties, memory loss, and paralysis. An electroencephalogram (EEG) is a tool that may detect anomalies in brain electrical activity, including those induced by a stroke. Using EEG data to determine the electrical action in the brains of stroke patients is an effort to measure therapy. Hence in this paper, deep learning assisted gene mutation analysis (DL-GMA) was utilized for classifying poststroke epilepsy in patients. This study suggested a model categorizing poststroke patients based on EEG signals that utilized wavelet, long short-term memory (LSTM), and convolutional neural networks (CNN). Gene mutation analysis can help determine the cause of an individual's epilepsy, leading to an accurate diagnosis and the best probable medical management. The test outcomes show the viability of noninvasive approaches that quickly evaluate brain waves to monitor and detect daily stroke diseases. The simulation outcomes demonstrate that the proposed GL-GMA achieves a high accuracy ratio of 98.3%, a prediction ratio of 97.8%, a precision ratio of 96.5%, and a recall ratio of 95.6% and decreases the error rate 10.3% compared to other existing methods.

## 1. Introduction

One of the most common causes of epilepsy is a stroke. For example, blood circulation to the brain may be disrupted, leading to a stroke [1]. Stroke symptoms include difficulty communicating, breathing, and comprehending and facial, arm, or leg numbness or paralysis. One of the long-term effects of a stroke is losing the ability to speak or understand or recall [2]. Patient populations with poststroke epilepsy (PSE) will rise in line with the aging population [3]. As a result of PSE, stroke patients' quality of life was severely lowered, and their families' responsibilities were greatly raised. Poststroke refers to how stroke patients find themselves after the occurrence [4]. Those who have had a stroke require rehabilitation to rehabilitate their bodies and reduce their impairments [5]. In addition to therapy, physical, cognitive, and mental rehabilitation is offered. However, determining the next therapy step requires regular monitoring and assessment [6]. Small blood veins in the brain, especially the cerebral vessels, are affected by this disorder, which reduces blood flow. Symptoms of CADASIL include migraines, numerous strokes, and dementia. In addition to these physical symptoms, patients may have cognitive decline, seizures, visual issues, and psychological issues such as severe depression and behavioral and personality disorders. Several devices may identify strokes: CT scan, MRI, EEG, and EMG. An initial diagnosis may be made with a CT scan or an MRI. EMG may be used for neurorehabilitation [7]. Recordings from EEG equipment may be used to facilitate the identification and monitoring of various forms of neurological rehabilitations [8]. It is vital to interpret EEG to correctly educate patients about their brain's status, explore whether stroke patients may utilize brain-computer interface (BCI), and extract relevant factors [9]. EEG is advantageous because it is inexpensive and poses a minimum danger to patients [10]. EEG equipment's noninvasive, elevated, user-movable, and cost-effectiveness make it a popular choice for capturing brain signals in BCI systems.

RETRACTED

For every gene, there is a unique variation in the DNA sequence. Because alterations in DNA do not necessarily result in illness, the word “gene variant” has replaced the term “gene mutation” as the more appropriate description [11]. Stroke-risk genes have been difficult to identify due to a lack of similar patient groups. Mendelian illnesses with distinct stroke-like characteristics have been investigated as genetic models for the more general population [12]. Other nonmodifiable risk factors for stroke, such as parental and family history, raise the risk. Genes linked to stroke may be discovered in two ways: through candidate gene analysis or genome-wide association (GWA) studies [13]. Genome-wide association studies (GWAS) aid researchers in discovering the genes responsible for a certain illness (or another trait). When examining the full collection of genetic material (the genome) of a large number of individuals, this technique looks specifically for some genetic changes known as single nucleotide polymorphisms or SNPs. Genetic factors for stroke include genes that encode proteins implicated in lipid metabolism, atherosclerosis, and thrombosis [14]. Using the GWA, which involves genotyping tens of thousands of different genetic variations, it is possible to discover new risk factors for stroke and new information on avoiding it [15]. No physiologically plausible gene or gene annotation can be found in the areas of interest; hence, GWA interpretation is left unclear [16].

Using the deep learning approach, computational computing is more efficient and permits for a more complicated feature extraction layer and processing of huge datasets and learning without supervision [17]. RNN and CNN are two popular approaches to deep learning that are often employed. CNN may be used for one-dimensional time series data types. This kind of neural network may interpret signals or sequentially store data. To make memory usage more realistic, data processing using recurrent neural networks must be classified as data that can be processed and data that cannot be handled, like LSTM. A preceding study found that RNN and LSTM may be utilized to identify strokes, diagnose epilepsy, and visualize motor images in stroke patients [18]. This study describes the localization of their stroke, specifies their risk factors, defines their genetic mutations, and correlates parameters to evaluate their importance in the tendency of stroke in older adults. RNN is a strong and extensively used machine learning and genomics approach. This study aims to examine RNNs with hidden long short-term memory (LSTM) units. LSTMs will be tested to discern patterns in the multilabel categorization of cerebrovascular signs or stroke.

RETRACTED

The main contributions of the paper are the following:

- Designing the deep learning assisted gene mutation analysis (DL-GMA) for detecting poststroke epilepsy in patients
- Introducing CNN and LSTM for predicting and classifying poststroke epilepsy from EEG signals
- The experimental results have been executed, and the suggested DL-GMA improves the accuracy, prediction, and low error rate compared to other existing methods

The rest of the study is structured as follows: Sections 1 and 2 discuss the introduction and related works on poststroke epilepsy. In Section 3, the DL-GMA has been proposed. In Section 4, results and discussion have been presented. Finally, Section 5 concludes the research article.

## 2. Related Works

Kazuki Fukuma et al. [18] introduced the PSSPECT for visualizing long-lasting hyperperfusion in poststroke epilepsy. Extensive and deep-seated distributions of postictal hyperperfusion were detected by subtracting postictal from the interictal SPECT. Subtraction SPECT was used to examine postictal hyper per fusion's lateral and regional distribution concerning stroke lesions, seizure symptoms, and epileptiform EEG results. An 86% increase in hyperperfusion was seen on subtraction SPECT in 43 of the 50 patients, while epileptiform EEG was found in 26 of the 50 patients (52%). Extending postseizure hyperperfusion was seen despite an average time gap of 19.1 hours between seizures and postseizure SPECT (median: 2.2-112.5 h).

Esmeralda C et al. [16] recommended the wavelet and convolutional neural networks (WCNN) to determine poststroke EEG signals. Using wavelet, a feature of machine learning, poststroke patients' EEG signals are analyzed for information. There are six different waves included in this feature: the delta, alpha, beta, theta, and mu waves. The EEG signal's five waves and amplitude properties are included in the model as a final touch. Findings from this study demonstrated that differentiating features need feature configuration. Amplitude and beta characteristics improved testing accuracy by 90 percent compared to 70 percent without these two elements. According to the experimental findings, the adaptive moment estimation (Adam) optimization model was also shown to be more stable than the stochastic gradient descent (SGD). In contrast to Adam, SGD may provide better results.

RETRACTED

Wanodya Sansiagi et al. [19] suggested the recurrent neural networks and long short-term memory (RNN-LSTM) for post-stroke detection of EEG signals. Patients were divided into “No Stroke” and “Stroke” for identification purposes. The waves that define a stroke are extracted from EEG signals via wavelet filtering. The identifying model's four waveforms and average magnitude are significantly impacting. In addition to SGD and adaptive moment optimization (Adam), various weight modification strategies were used in the research. According to this study, wavelets without amplitude characteristics had an accuracy of 94.80 percent for fresh information using the Adam model. SGD and Adam, the optimization models utilized in this work, have a precision difference of 94.8%.

Haim Golan et al. [20] proposed HyperBaric Oxygen Therapy (HBOT) using imaging-based predictors for poststroke patients. Hyperbaric sessions for all patients included 90 minutes of exposure to 100% oxygen at 0.2 MPa every day for 60 days. Patients' responses to therapy were compared to SPECT/CT-detected volume changes in the penumbra region around the stroke zone. During HBOT, the penumbra zone (363 ± 20.5 ml) was dramatically reduced in size in the patients who significantly improved their clinical neurologic condition and quality of life (*n* = 24). The patient's penumbra zone volume was only (148 ± 29.3 ml) in those who did not benefit from HBOT (*n* = 20), and its further reduction during HBOT was minimal. In 18 patients with penumbra volumes ranging from these two extremes, the HBOT findings were ambiguous. A broad penumbra region around the stroke zone may considerably predict better clinical outcomes after HBOT in poststroke patients, as these data confirm our theory. HBOT for stroke patients can advantage from a SPECT/CT-based evaluation of the penumbra volumes, which may be used as a selection tool.

RETRACTED

Shujun Zhang et al. [21] recommended that DNN with massive data learning ability supplies a powerful tool for stroke lesion detection. More than 5,000 MRI images of 300 ischemic stroke patients were utilized to study the features of stroke lesions and identify them using sophisticated automated techniques. Professional physicians meticulously designated each lesion location in these images for credibility and efficacy. 89.77 percent accuracy in automated lesion diagnosis is achieved by combining Faster R-CNN, YOLOV3, and SSD deep learning object detection networks. There is also a good statistical study of lesions and probable illnesses concerning their locations and forms. Intelligently aided diagnosis, prevention, and treatment of ischemic stroke are possible because of this study's findings.

Based on the survey, there are several challenges in existing models, such as postictal subtraction single-photon emission computed tomography (PSSPECT), recurrent neural networks, long short-term memory (RNN-LSTM), wavelet and convolutional neural networks (WCNN), and HyperBaric Oxygen Therapy (HBOT) in achieving high accuracy, prediction, and low error rate. Thus, the DL-GMA has been suggested in this post. DL-GMA is discussed in the next section concisely.

## 3. Deep Learning-Assisted Gene Mutation Analysis (DL-GMA)

A blood vessel blockage or burst causes the blood supply to the brain to stop, resulting in a stroke. It may be caused by plaque accumulation in the brain or hypertension in the individual. Dementia, aphasia, and blurring of vision are all possible side effects of a stroke. A new model was developed to predict stroke based on DL using the raw and distinctive values of EEG acquired in real-time. The suggested system is a collection of (i) a model that gathers data, (ii) a model that transfers the produced biological signal to servers, (iii) a model that examines the stored biological information and then extracts and handles frequency attribute, (iv) a DL-based learning and forecasting modules based on LSTM and CNN networks, (v) biological-signal-based strokes forecasting model, and (vi) gene mutation analysis. Pretreatment procedures and characteristics like electrocardiogram (ECG) and electroencephalogram (EEG) information from older persons are then extracted and stored by the initial system. This is based on biological signal data. Finally, bio-signal information is employed as input for the DL model to forecast and assess poststroke abnormalities in elder persons.

Figure 1 shows the proposed DL-GMA. This study used bio-signal data as input, such as electroencephalography (EEG) signals to classify and predict stroke illnesses utilizing bio-signals. However, every bio-signal information was captured in real-time. Once the device is set up, six channels of EEG information are gathered at a sample ratio of 1 kHz, and the frequency attribute value is mined from the raw data. Among the extracted frequency feature value, the power values, which express the degree to which every frequency element has seemed, and comparative values, which denote the relative fraction of every frequency element in the frequency domain for all regions, are of high significance. An LSTM and CNN can be described by adding convolutional neural network layers on the front end, trailed by long short-term memory layers with a dense layer on the outcome of stroke image classification.

RETRACTED

Figure 2 shows poststroke epilepsy images. The picture data are collected from https://radiopaedia.org/ [22]. For the training and testing phases, 100 digital pictures were used, including 40 photos of ventricular tachycardia stroke, 40 images of cardiogenic shock, 10 images of the common brain, and 10 images of functional brain for the validation data. The Skull and spinal cord abnormalities may be found with a head MRI and determine whether a stroke is ischemic or hemorrhagic. CNN and LSTM are widely used for image processing. Features are automatically extracted from CNN's hidden layers, and deep network models generally corroborate the health of the features they discover. Stroke is connected with various genetic mutations, many of which act in concert rather than as discrete genes. Strokes in older persons with genetic abnormalities should be recognized to begin aggressive anticoagulation, warn patients about their risk of stroke, provide information on other risk factors, and discuss the prognosis. EEG recordings train convolutional neural networks (CNNs) to identify seizures. The convolution method is performed by each electrode signal being convolved with Kernel functions, which are single-dimensional filters used to extract the temporal information from recorded EEG signals, and then further supplied from the output functions to build feature maps. The pooling layer follows the output function of the rectifier linear unit (ReLU). In the end, features are transmitted from completely linked hidden layers of information. The softmax function has been used to map between “0” and “1”.

### 3.1. Stage 1: Wavelet Extraction

This study evaluates an electroencephalogram (EEG) feature extraction model based on the multiresolution wavelet transforms. The wavelet technique is usually utilized to preprocess signal processing, noise reduction, and image processing, which gives excellent outcomes. The breakdown into a frequency element and subsequent reconstruction into the period domain are included in a wavelet. Thus, an EEG signal that is nonstationary can be examined utilizing wavelet. Decompositions have two procedures that are convolutional and down-samplings. Discrete wavelet conversions of signals *y*(*m*) are provided by decompositions *D*(*ρ*, *τ*) in

(1) $$\begin{array}{c} D\left(\rho ,\tau \right)=\underset{m}{\sum }y\left(m\right)\varphi_{\rho ,\tau }\left(m\right). \end{array}$$

And reconstruction is done:

(2) $$\begin{array}{c} \hat{y}\left(m\right)=\underset{\rho }{\sum }\underset{\tau }{\sum }D\left(\rho ,\tau \right)\varphi_{\rho ,\tau }\left(m\right). \end{array}$$

As shown in (1) and (2), where *φ*(*m*) is the wavelet family.

(3), consisting of *ρ* and *τ* are scale and shift factors, is a basic wavelet function.

(3) $$\begin{array}{c} \varphi_{\rho ,\tau }\left(m\right)=\frac{1}{\sqrt{\left|\rho \right|}}\varphi \left(\frac{m-\tau }{\rho }\right). \end{array}$$

Every decomposition stage creates approximation signals as partial low-frequency bands and information like high-frequency filters. The low coefficient or the approximation and high feature coefficient are determined utilizing equations (4) and (5), where *f*(*m*) and *h*(*n*) are the high pass and low pass filters, correspondingly. Different practices of a wavelet function containing Symlet2 comprise four coefficients. Signal decomposition takes numerous stages to generate beta, alpha, delta, theta, and mu waves.

(4) $$\begin{array}{c} \text{Approximation }x\text{ low }\left[l\right]=\underset{m}{\sum }y\left[m\right].h\left[2l-m\right], \end{array}$$

(5) $$\begin{array}{c} \text{Detail }x\text{ high }\left[l\right]=\underset{m}{\sum }y\left[m\right].g\left[2l-m\right]. \end{array}$$

As inferred from equations (4) and (5), where *i* and *l* are integers that specify the scaling and dilatation of the basis function. It is based on the shapes or positions of the signal. *l* indicates *l* train data, *m* is a feature for each training data, *y*(*n*) denotes *Mth* feature or original signal, *h*(*m*) indicates low-pass filter coefficient, and *g*(*m*) denotes high-pass filter coefficients. The next stage explains the CNN model for processing extracted EEG features.

RETRACTED

### 3.2. Stage 2: Convolutional Neural Network (CNN)

The convolutional neural network can classify poststroke images effectively. CNN can handle data in the temporal domain, such as EEG data. Extracting EEG features that match a classification variable is critical in pattern recognition. It has been shown that strokes may be prevented or reduced by employing the symmetrical brain index and relative frequency band ratio and the various bands' amplitude and rhythm research. Features are extracted using convolution and classification, respectively, in a CNN. Once this layer is trained, it will be used to create a feature used in the CNN identification layer. It is possible to adjust weights in learning by using stochastic gradient descent (SGD) or adaptive moment estimation (Adam). Adaptive backpropagation is utilized for BCI, and AdaDelta follows a similar approach.

Figure 3 shows the CNN architecture. Convolution contains neurons organized to have the pixel length that makes up kernels. The kernel transfers as much as the stride values to the right until the finish. The convolutional step must identify the activation values utilized for the contents of kernels. To determine output values by dots product among input and outcome of kernels to generate an output termed feature maps (FMs) utilizing (6) as operators.

(6) $$\begin{array}{c} FM\left(n\right)=\underset{c_{1}=0}{\sum }C\left(c_{1}\right)*J_{\left(c_{1}+i_{1}\right)}. \end{array}$$

As discussed in (6), where *FM* is feature maps, *J* denotes input, *C* indicates convolution filters, *c*_*j*_ is column indices of *j* filters, *n* denotes feature maps number, and *i*_1_ indicates feature maps columns.

The convolution among the signal and kernels shifts as much as the stride values in this layer. It identifies the next output dimensions. While zero-padding identifies the number of auxiliary values for 0 intensity in the adjacent region or input sides, get map features can be shown in

(7) $$\begin{array}{c} \text{output}=\frac{S-F-2P}{W}+1. \end{array}$$

As shown in (7), *S* denotes weight, F is a convolution function, and *P* is a probability rate. If signals are convoluted with stride one, there is a right shift of one point.

Rectified Linear Unit (ReLU) is the activation progression function to remove negative values to 0, and activation function *y* is called

(8) $$\begin{array}{c} f\left(y\right)=\max\left(0,y\right). \end{array}$$

The step of max pooling feature maps creates a minimum size by decreasing and does not remove the leading feature by taking the maximum values from the activation outcomes. This research obtains a pooling distance of 2*x*1 pixels to 1*x*1 pixels.

Temporarily, the softmax activation functions are utilized at output layers to compute the likelihood of every destination class and select the biggest one utilizing

(9) $$\begin{array}{c} x_{Yj}=\frac{e^{y^{Q}y_{j}}}{\sum_{i=0}^{l}e^{y^{Q}y_{j}}}. \end{array}$$

Subsequently, the cross-entropy activation functions, entitled loss functions, calculate the deviation among targets and outputs from the feedforward calculation. The cross-entropy functions can be demonstrated in

(10) $$\begin{array}{c} \text{Loss}\left(W,K\right)=-\underset{j}{\sum }K_{j}\log\left(W_{j}\right). \end{array}$$

As inferred from the (10), *W* is a softmax function and *K* is the convolutional kernel. The next stage defines the LSTM network for classifying stroke images.

RETRACTED

### 3.3. Stage 3: Long Short-Term Memory (LSTM)

The existing recurrent neural network is a kind of artificial neural network wherein data persist inside the NN, and it has been utilized for automatic translation, image description generation, etc. The recurrent neural network has the disadvantage that as the duration of the input series increases, the reduction in slopes causes its learning capacity to diminish gradually. To address these issues, this study uses the LSTM models, which augment cell states to the hidden states of the recurrent neural network. The forget gate *f*_*t*_ denote gates for forgetting historical data inside an NN, which conserves the data completely if the formula outcome is one and removes it if it is zero.

(11) $$\begin{array}{c} f_{t}=\rho \left(S_{f}\cdot \left[g_{t},y_{t}\right]+a_{f}\right). \end{array}$$

As shown in (11), *f*_*t*_ denotes forget gates, *S*_*f*_ denotes weight function, *g*_*t*_  indicates the hidden gate, *a*_*f*_  denotes bias function, and *y*_*t*_ is the input gate. The input gate for recalling the current data within an NN, where new info is stored in cell states, may be identified. Initially, expression (12) identifies which values to update and then arranges to augment the novel candidate value, the ${\hat{C}}_{t}$ vectors, to cell states via expression (13). The state can be said to be equipped by uniting the two datasets from expression

(12) $$\begin{array}{c} j_{t}=\rho \left(S_{j}\cdot \left[g_{t-1},y_{t}\right]+a_{j}\right),\\ {\hat{C}}_{t}=\tanh\left(S_{C}\cdot \left[g_{t-1},y_{t}\right]+a_{C}\right). \end{array}$$

It then updates the preceding states, *C*_*t*−1_, to make novel cell states, *C*_*t*_.

Figure 4 shows the LSTM model. LSTM is utilized to conquer the amount of information as the gate process progresses. Long short-term memory has a standard unit termed memory blocks inside the hidden layer. This notion is an additional way to compute hidden states. The term “cell” refers to the temporary storage of information in a memory block. Long short-term memory inputs are taken from the first states *g*_*t*−1_ and present inputs *y*_*t*_. As shown in Equation (13), the prior state is multiplied by ft, while forgetting in the initial phase selects what is forgotten and accumulates $j_{t}*{\hat{C}}_{t}\text{.}j_{t}*{\hat{C}}_{t}\;$ is a value that improves or decreases depending on the number of values to be updated.

(13) $$\begin{array}{c} C_{t}=f_{t}*C_{t-1}+j_{t}*{\hat{C}}_{t}. \end{array}$$

In conclusion, the output gates *o*_*t*_ obtain how much data are signified inside the NN, where the outcome is strained based on cell states. The cell states are input into the *tanh* layers to get values between −1 and 1. These values are multiplied by the outcome of the formerly computed sigmoid gates, which permits only required parts to be articulated as an outcome. This progression is demonstrated in

(14) $$\begin{array}{c} o_{t}=\rho \left(S_{o}\left[g_{t-1},y_{t}\right]+a_{o}\right),\\ g_{t}=o_{t}*\;\tanh\left(C_{t}\right). \end{array}$$

The stroke image has been identified and classified using the LSTM network. The following stage discusses the gene mutation analysis of poststroke epilepsy effectively.

RETRACTED

### 3.4. Stage 4: Gene Mutation Analysis

The stroke risk has been analyzed using CT, MRI, carotid ultrasound, and echocardiogram. Ischemic stroke warning signs may appear as early as seven days before an attack, and quick treatment is needed to avoid serious brain damage. Symptoms such as a headache, numbness, or tingling might occur many days before a major stroke in some individuals. Study participants who had mini-stroke symptoms up to a week before their stroke had a 43% chance of having a major stroke. In this study, researchers analyzed where the stroke occurred, the risk factors, and how the genetic abnormalities affected their vulnerability to stroke. The frequency of gene mutations in the four types of lesions has been examined using Chi-square testing (cerebral venous, cerebral arterial, spinal, and minor vessel disease). Study participants were compared to those with mutations in the MTHFR (mutations C677 T and A1298 C) and Factor V (FV) genes. The four-stroke types were subjected to a 4-sample test to ensure proportional equivalence. Finding possible genetic factors of stroke risk is difficult due to a lack of comparable patient groups. Mendelian diseases with distinct stroke-like symptoms have been used as genetic models for the general population. Most strokes are arterial and linked largely with the Factor V and MTHFR gene mutation described in Table 1.

Figure 5 shows the gene mutation of poststroke and central pain detection. Neuronal excitability may rise due to morphological, neurochemical, excitotoxic, and inflammatory alterations in the central nervous system (CNS). A loss of inhibition and an increase in facilitation may lead to central sensitization and persistent pain. For the healing of central pain, pharmacological medications may reduce neuronal hyperexcitability, which supports this theory. Neurotransmitters in the hypothalamus or the cortical that spontaneously discharge may be linked to regional poststroke pain (CPSP). (A) Whenever the SpinoThalamic Tract (STT) connection towards the downstream laterally hemisphere is removed, the medial thalamus is disinhibited. (B) The hypothesis of thermosensory disinhibition. This disinhibition of medial limbic networks, which includes the parabrachial nucleus, periaqueductal grey, and anterior cingulate cortex, is caused by a lesion in the left-to-right cool-signaling spinothalamocortical projections to the insula via the posterior portion of the ventral medial nucleus (ACC). (C) For example, pain results when neospinothalamic, lateral, or medial STT projections lose the usual reserve from the fast-conducting neospinothalamic or lateral STT projection. (D) When calcium spikes at a low threshold induce hyperactive bursts in the thalamus, this might lead to central discomfort. (E) The theory of dynamic reverberation. When the STT is disrupted, central pain is caused because the usual oscillatory conversation between the cortex and thalamus has been disrupted.

RETRACTED

## 4. Results and Discussion

This study proposed DL-GMA for poststroke epilepsy prediction and classification. The image data were acquired from https://radiopaedia.org/ [21]. Radiopaedia.org is an open-edit radiological resource that is quickly expanding and is being produced by radiologists and other health professionals from all around the world. Radiology papers and cases may be found in abundance at Radiopaedia. Ideally, one should use various resources best suited to their specific demands regarding the accuracy and medical image quality. Each patient case is owned by a contributing member, after which it may be seen and contributed to articles or playlists by the community. Dedicated editors ensure that the content adheres to quality standards and addresses any privacy issues. The test datasets use 100 pictures and videos of hyperacute and myocardial infarction (mi, ten photos of the functional brain, and ten images of the functional brain for the trained data and evaluating databases, respectively). This paper discusses the accuracy ratio, prediction ratio, precision ratio, recall ratio, and the error rate for comparative analysis.

### 4.1. Accuracy Ratio

A stroke, often known as a brain attack, may be caused by a ruptured or clogged artery. It is possible to have a stroke or a brain attack when one or more blood arteries in the brain burst or if anything prevents blood flow to a particular location. Because stroke illness is becoming more prevalent globally, especially among those with lower incomes and older individuals, healthcare services are in critical need of a solution that would assist them in reliably and rapidly diagnosing stroke disorders at a reasonable cost. The preliminary findings indicate that the raw data on their own might be used to make accurate predictions about stroke illness. A comparison of the prediction accuracies of CNN and LSTM is being made to discover which kind of DL models are most appropriate for starting working EEG information. The accuracy ratio has been determined by (5) and achieves a high accuracy ratio of 98.3%.  Figure 6 demonstrates the accuracy ratio.

RETRACTED

### 4.2. Prediction Ratio

A seizure may be brought on by a rapid increase in aberrant brain electrical activity, which disrupts the messages sent to the nerves. Stroke damage in the brain may create this electrical disruption. Antiepileptic medicines (AEDs, often known as anticonvulsants), vagus nerve stimulation, or surgery are commonly used to treat poststroke epilepsy. Several AEDs may help manage poststroke epilepsy by reducing seizure frequency and intensity. The raw EEG data collected in this study may be used to create a real-time stroke risk prediction system. Stroke disease may be predicted using a variety of biological signals, including images. CNN and LSTM analyze real-time brainwave data to forecast strokes based on the characteristics learned from the offline processing unit. Brain activity may be measured using an EEG and help determine the cause of various diseases, including epilepsy and other seizures. Small metal discs (electrodes) placed on the scalp are used to assess electrical activity in the brain during an electroencephalogram (EEG). Medical professionals may then use these data to treat patients better. Medical professionals may use this information to anticipate strokes better and provide a timely and accurate diagnosis. The prediction ratio has been identified using (6).  Figure 7 shows the prediction ratio.

### 4.3. Precision Ratio

According to this definition, the precision rate is the proportion of people who have had a stroke out of those who have had a favorable experience. Precision and recall are beneficial where the number of observations fitting one class is suggestively lower than those fitting the other classes in poststroke epilepsy detection. These metrics are, thus, used in the evaluation of pixel-wise classification, where the number of pixels corresponding to each class varies considerably.

(15) $$\begin{array}{c} \text{Precision}=\frac{TP}{TP+FP}. \end{array}$$

As shown in (15), TP denotes true positive and FP indicates false positive. The proposed AI-SLDCM model enhances the precision ratio by 96.5%.  Figure 8 illustrates the precision ratio.

RETRACTED

### 4.4. Recall Ratio

There has been an increase in recent years in the occurrence of stroke misdiagnosis, particularly in the failure to identify stroke (stroke chameleon [SC], false negative) and the overdiagnosis of stroke (stroke mimic [SM], false positive). The F1 score is an equivalent weighting of the precision and recall and quantifies how well the model performs in general. The recall measures the ability to perceive the occurrence of a class, which is a given stroke image.

(16) $$\begin{array}{c} \text{Recall}=\frac{TP}{TP+FN}. \end{array}$$

As shown in expression (18), TP denotes true positive and FN indicates false negative. The proposed AI-SLDCM model enhances the recall ratio by 95.6% compared to other existing models.  Figure 9 signifies the recall ratio.

### 4.5. Error Rate

Stroke misdiagnosis may be defined as a failure to detect a stroke immediately after or while it is occurring or noticing signs of an impending stroke. This study discusses the frequency of stroke misdiagnosis and obtains stroke subgroup at great risk for particular diagnostic mistakes. Policies to reduce diagnostic mistakes in stroke have mainly concentrated on early stroke identification through bedside inspection policies and clinical decision rules. Adam is a deep learning approach that calculates the amount of distinct learning for every variable to adaptively decrease the chance of error in stroke classification. Increasing the weight of each training session may be accomplished in several ways. It is possible that certain approaches optimize for convergence and create errors fast or have minimal cross-entropy values. Adam's model is unstable because of the rapid decrease in errors and has quick convergence features. Adaptive moment estimation is a model for the optimization method for gradient descent. The technique effectively works with a significant issue, including any information or variables. It needs less memory and is effective. The challenge of utilizing learning rate plans is that their hyperparameters have to be described in advance, and they depend profoundly on the type of model and issue. Another difficulty is that the same learning ratio is employed for all variable updates. The less error rate is determined using (8).  Figure 10 shows the error rate.

The proposed DL-GMA achieves high accuracy, prediction, precision, recall ratio, and low error rate compared to other existing methods, PSSPECT, WCNN, RNN-LSTM, and HBOT.

## 5. Conclusion

This paper presents the DL-GMA for poststroke epilepsy prediction and classification. The parameter analysis is used to evaluate the accuracy of the series of features input into the CNN and LSTM learning models. Initially, it was assumed that the search for a novel or undiscovered genes that may open up new treatment pathways for brain destruction or protection was driving the search for differential gene expression. The convolutional neural network may assist neurologists in identifying stroke based on the results of the classification of stroke from head scan images. EEG signals utilizing wavelet, CNN, and LSTM data may be utilized to determine poststroke patients, as shown in this research. The outcomes of the tests utilizing raw data, power value, and relative value indicated that the best accuracy in stroke prediction was attained by using raw data. The simulation consequences show that the suggested GL-GMA attains a high accuracy ratio of 98.3%, a prediction ratio of 97.8%, a precision ratio of 96.5%, and a recall ratio of 95.6% and decreases the error rate by 10.3% compared to other existing methods. A predictive model for predicting the probability of stroke is obtained by training. Such a high prediction accuracy will help prevent the occurrence of a stroke. Gathering a dataset containing images like brain scans to forecast the likelihood of stroke would be more capable in the future. In the future, this study will use more risk factors to forecast deep learning methods and compare them to other approaches.

RETRACTED

## Figures and Tables

**Figure 1:** Proposed DL-GMA.

**Figure 2:** (a) No stroke. (b) Stroke. (c) Hyperacute stroke. (d) Ischemic stroke.

**Figure 3:** CNN architecture.

**Figure 4:** LSTM model.

**Figure 5:** Gene mutation of poststroke and central pain detection.

**Figure 6:** Accuracy ratio.

**Figure 7:** Prediction ratio.

**Figure 8:** Precision ratio.

**Figure 9:** Recall ratio.

**Figure 10:** Error rate.

**Table 1:** Pathologies linked with every gene mutation.

Gene	Pathology
MTHFR	Brain venous thrombosis and cerebral artery stroke
Factor V	Cerebral artery stroke and brain venous thrombosis

## Data Availability

The datasets generated during and/or analyzed during the current study are not publicly available due to sensitivity and data use agreement.
